The article "ANOVA-Based Analysis of Early Blood Transfusions on Hemodynamics with Severely Injured Trauma Using Bedside Ultrasound Imaging" was retracted in 2023. Reasons: signs of a paper mill; suspected computer-generated content; unreliable results or conclusions; lack of ethics approval or compliance.

# ANOVA-Based Analysis of Early Blood Transfusions on Hemodynamics with Severely Injured Trauma Using Bedside Ultrasound Imaging

**DOI:** 10.1155/2021/5263454

**Published:** 2021-07-22

**Authors:** Lei Song, Jianguo Zhang, Junliang Liu

**Affiliations:** Department of Intensive Care Unit, The Affiliated Qingdao Hospital of Shandong First Medical University, Qingdao 266109, Shandong, China

## Abstract

The focus of the study was to quantitatively analyze the influence of early massive blood transfusions (MBTs) on the hemodynamics and prognostic living quality of patients with severely injured trauma. 114 patients with severely injured trauma were enrolled into MBT group (67 cases) and nonmassive blood transfusions (NBT) group (47 cases) according to whether they accepted MBTs within 24 hours after the admission. All patients had bedside ultrasound technology scanning. Furthermore, the indexes were calculated for inferior vena cava (IVC), peripheral arteries, and heart. The prognostic deaths were recorded. It was found that, in the MBT group, the mortality was lower (7.55% vs. 24.23%) (*P* < 0.05), and these indexes were higher for the IVC expansion (IVCE), the respiration variation index (RVI) of IVC (ΔIVC_2_), the peak flow velocity RVI of brachial artery (ΔVpeak_BA_), femoral artery (ΔVpeak_FA_), left ventricular outflow tract (ΔVpeak_L_), and aorta (ΔVpeak_AO_), as well as peak flow velocity time integral RVI of aorta (ΔVTI_AO_) (*P* < 0.05). In conclusion, early MBTs can elevate survival rate and prognostic living quality and alleviate the atrophy degree of IVC, peripheral artery, and blood vessel of patients with severely injured trauma. Furthermore, bedside ultrasound scanning demonstrated superb capabilities in quantitatively displaying hemodynamics and outcomes of MBTs of patients with severely injured trauma.

## 1. Introduction

Trauma refers to the destruction of tissues or organs caused by mechanical factors. Due to the differences in injured parts, injured tissues, and skin integrity, the severity of trauma is also different [1, 2]. Among them, severely injured trauma may cause systemic reactions, with local manifestations such as pain, swelling, tenderness in the injured area, and even fatal symptoms such as hemorrhage, shock, suffocation, and disturbance of consciousness [3]. Relevant studies have reported that trauma has become the leading cause of death for people under the age of 40, even exceeding the total number of deaths from AIDS, tuberculosis, and malaria [4]. Furthermore, the people who die from trauma every year are mostly teenagers, which greatly affect social stability and economic development. Traumatic bleeding has always been the main cause of death in trauma patients. Clinical observations have revealed that, in addition to bleeding caused by liver and spleen lacerations and fractures, the abnormal coagulation function of patients is also a very key factor for continuous bleeding [5, 6]. At present, the clinical treatment methods of bleeding in patients with severely injured trauma mainly contain permissive hypotension, hemostasis, and resuscitation. Patients with heavy bleeding need timely blood transfusion therapy to correct coagulation disorders and improve the prognosis of trauma patients. Therefore, the primary objective of the study was to explore the influence of massive transfusions on patients with severely injured trauma.

With the advancement of imaging, there are various imaging examination methods used in clinical practice. However, being time-consuming, the routine imaging scan is not suitable for the diagnosis of trauma and bleeding patients, such as ultrasound, conventional CT, X-ray, and angiography [7]. Plain X-ray is the earliest imaging method used. It features simple operation and low price, but the display of soft tissue is poor, and it is prone to misdiagnosis and missed diagnosis [8, 9]. Angiography can be used to observe the blood flow in the arteries or veins of the head, arms, legs, chest, back, or abdomen, but it is easily affected by body movements. Although conventional CT is easy to operate, it cannot show minor damage [10]. As a result, bedside ultrasound has been a hotspot in clinical research in recent years. It is usually used in emergency and life-threatening conditions to speed up diagnosis and treatment [11]. Because bedside real-time ultrasound performs a single or local examination for a specific clinical phenotype, it greatly shortens the examination time and can quickly provide crucial information, such as the patient's systolic, diastolic function, volume load, heart structure, and hemodynamics. Balík [12] adopted transcranial Doppler ultrasound to monitor the cerebral blood flow of severely injured trauma patients. The results showed that ultrasound images can accurately diagnose the hemodynamics and position the blood vessels before intubation to avoid potential complications and unnecessary platelet transfusion. Gomora-García et al. [13] used ultrasound to guide the treatment of patients with painful shoulder trauma syndrome. The results found that ultrasound-guided treatment demonstrated better effects in contrast with conventional treatment and was safer. Therefore, the further aim was to apply bedside ultrasound to analyze the diagnostic results of severely injured trauma.

In summary, bedside ultrasound demonstrated superb capabilities in clinical diagnosis and treatment of severely injured trauma patients. Based on this, 114 patients with severely injured trauma were enrolled into MBT group (67 cases) and NBT group (47 cases) according to whether they accepted MBTs within 24 hours after the admission. All patients had bedside ultrasound technology scanning. Furthermore, the indexes were calculated for IVC, peripheral arteries, and heart, to quantitatively analyze the influence of early MBTs on the hemodynamics and prognostic living quality of patients with severely injured trauma.

## 2. Materials and Methods

### 2.1. Selection of Samples

114 patients with severely injured trauma, who were admitted to the hospital between November 25, 2017, and February 10, 2020, were selected for analysis, with an average age between 20 and 67. All of them had bedside ultrasound scanning. The study has been approved by the Medical Ethics Committee of the hospital. The patient and his/her family members have been informed of the study and signed the consent letters.

Inclusion criteria: (i) patients older than 18 years; (ii) patients who underwent bedside ultrasound within 12 hours after trauma; (iii) patients with an abbreviated injury scale (AIS) score greater than 3; (iv) patients who can cooperate with the doctors.

Exclusion criteria: (i) patients with unstable hemodynamics; (ii) patients with congenital heart disease; (iii) patients with severe kidney disease; (iv) patients with aortic and great vessel split; (v) patients with incomplete clinical data; and (vi) patients with head trauma.

### 2.2. Grouping of Subjects

114 patients with severely injured trauma were enrolled into MBT group (67 cases) and NBT group (47 cases) according to whether they accepted MBTs within 24 hours after the admission. The standard of massive blood transfusions no less than 20 U red blood cells were injected within 24 hours after admission.

### 2.3. Bedside Ultrasound Scanning

Patients accepted bedside ultrasound scanning before and after treatment by Sono ultrasonic machine (USA). A 2.5 MHz heart probe was used. The patient was in a supine position. The long axis of the left heart next to the sternum was selected, that is, the long axis of the left ventricle. The heart probe was placed between 3 and 4 intercostals of the left edge of the sternum. The detection direction was parallel to the right sternoclavicular joint to center the transverse section of the thoracic aorta. The probe was slightly upward on the basis of the four-chamber heart at the apex of the heart, and the scanning plane passed through the aortic root to obtain the transverse section of the aortic root, the longitudinal section of the left ventricle, the longitudinal section of the right atrium, the longitudinal section of the right ventricle, and the longitudinal section of the right atrium, namely, the image of the five-chamber heart at the apex. IVCE, ΔIVC_2_, ΔVpeak_BA_, ΔVpeak_FA_, ΔVpeak_L_, ΔVpeak_AO_, and ΔVTI_AO_ were recorded. IVCE refers to the difference between the maximum diameter (IVC_max_) and the minimum diameter (IVC_min_) of IVC at 2 cm of the opening of right atrium which was then divided by IVC_min_. The equation is as follows:

(1) $$\begin{array}{c} \text{IVCE}=\frac{{\text{IVC}}_{\text{max}}-{\text{IVC}}_{\text{min}}}{{\text{IVC}}_{\text{min}}}\times 100\text{\%.} \end{array}$$

### 2.4. Statistics

The data were processed by SPSS19.0. The mean ± standard deviation ($\bar{x}$ ± *s*) illustrated how to calculate the measurement data. Count data were expressed as a percentage (%). Age, BMI, length of hospital stays, male-female ratio, and mortality were compared using independent *t*-test. The analysis of variance was applied to compare indexes for IVC, peripheral arteries, and heart. *P* < 0.05 indicated statistically significant differences.

## 3. Results

### 3.1. Comparison of Basic Data

Figures 1 and 2 show the comparison of basic data of patients. In the MBT group, the patients were 43.51 ± 9.73 years old, their BMIs were 24.76 ± 4.79 m^2^/kg, the ratio of males was 68.56%, and the length of hospital stay was 33.51 ± 7.53 days. In the NBT group, the patients were 41.73 ± 11.24 years old, their BMIs were 26.11 ± 5.22 m^2^/kg, the proportion of males was 64.37%, and the length of hospital stay was 31.75 ± 8.22 days. There was no notable difference in age, BMI, the ratio of males, and the length of hospital stays (*P* > 0.05).

Figure 3 shows traumatic kidney injury in a male patient (aged 34 years old) caused by a car accident. It was evident that the lower part of the right kidney was morphologically abnormal, there was a heterogeneous echogenic mass, and an acoustic image of a clot can be seen in the bladder.  Figure 4 shows traumatic renal parenchymal laceration caused by a car accident in a female (aged 26 years old). The renal parenchymal laceration with hematoma was visible, the renal capsule was intact, and a hypoechoic mass was seen in the middle parenchyma with a clear boundary.

### 3.2. Comparison of Mortality

Figure 5 shows the comparison of mortality of the two groups. It was evident that, in the MBT group, the mortality was lower (7.55% vs. 24.23%) (*P* < 0.05).

### 3.3. Comparison of IVCE and IVC_2_

Figure 6 shows the comparison of IVCE and IVC_2_. It was evident that, in the MBT group, IVCE (21.54 ± 4.11 vs. 13.52 ± 3.27) and IVC_2_ (13.52 ± 3.27 vs. 13.17 ± 2.86) were obviously higher (*P* < 0.05).

### 3.4. Comparison of ΔVpeak_L_

Figure 7 shows the comparison of ΔVpeak_L._ It was evident that, in the MBT group, ΔVpeak_L_ was obviously higher (19.56 ± 2.76 vs. 14.11 ± 1.85) (*P* < 0.05).

### 3.5. Comparison of ΔVpeak_AO_ and ΔVTI_AO_

Figure 8 presented the comparison of ΔVpeak_AO_ and ΔVTI_AO._ It was evident that, in the MBT group, ΔVpeak_AO_ (15.77 ± 1.48 vs. 12.75 ± 1.51) and ΔVTI_AO_ (18.88 ± 1.62 vs. 13.47 ± 1.36) were obviously higher (*P* < 0.05).

### 3.6. Comparison of ΔVpeak_BA_ and ΔVpeak_FA_

Figure 9 shows the comparison of ΔVpeak_BA_ and ΔVpeak_FA._ It was evident that, in the MBT group, ΔVpeak_BA_ (21.55 ± 1.42 vs. 14.92 ± 1.36) and ΔVpeak_FA_ (17.53 ± 1.38 vs. 13.66 ± 1.51) were obviously higher (*P* < 0.05).

## 4. Discussion

Patients with severely injured trauma should see a doctor in time to determine the degree of trauma as quickly as possible, so as to provide targeted clinical treatment. Although the domestic diagnostic technology has been greatly improved in recent years, the shock and mortality caused by severely injured trauma are still high, so it is very important to adopt effective diagnostic methods [14, 15]. In the study, bedside ultrasound scanning was applied to patients to analyze the influence of early MBTs on hemodynamics and prognostic living quality of them. It was found that, in the MBT group, the mortality was lower (7.55% vs. 24.23%) (*P* < 0.05). This was in line with the research results of Nolte et al. [16]. Existing research believes that early MBTs for severely injured trauma can actively improve the coagulation disorder after acute trauma, thereby enhancing the prognosis of trauma patients. It suggested that early MBTs can elevate survival rate and prognostic quality of patients and reduce shock death. In the MBT group, IVCE (21.54 ± 4.11 vs. 13.52 ± 3.27) and IVC_2_ (13.52 ± 3.27 vs. 13.17 ± 2.86) were obviously higher (*P* < 0.05). This was inconsistent with the research results of Cui and Wu [17]. IVC is the main blood vessel that returns blood to the abdominal organs and lower limbs. In the early stage of trauma, the internal diameter is reduced due to the reduction of blood flow back to the lower limbs and abdomen. However, early MBTs can effectively compensate for the ischemic state of patients with severely injured trauma and improve IVCE and IVC_2_.

In the MBT group, ΔVpeak_L_ was obviously higher (19.56 ± 2.76 vs. 14.11 ± 1.85) (*P* < 0.05). This was different from the research results of Endo et al. [18], which may be because of the different sample sources. It demonstrated that MBTs allow the patient to receive enough blood to restore normal blood flow. In the MBT group, ΔVpeak_AO_ (15.77 ± 1.48 vs. 12.75 ± 1.51) and ΔVTI_AO_ (18.88 ± 1.62 vs. 13.47 ± 1.36) were obviously higher (*P* < 0.05). This illustrated that the early MBTs greatly affected the abdominal aortic vessels, which may be due to the fact that the abdominal aortic vessels mainly regulate blood flow through changes in tube diameter and distal resistance and will supplement the overall capacity of human body by reducing its own blood flow when there is trauma [19]. In the MBT group, ΔVpeak_BA_ (21.55 ± 1.42 vs. 14.92 ± 1.36) and ΔVpeak_FA_ (17.53 ± 1.38 vs. 13.66 ± 1.51) were obviously higher (*P* < 0.05). This was aligned with the research results of Roden-Foreman et al. [20]. Arteries transport blood rich in oxygen and various nutrients to various parts of the body, while severely injured trauma can cause abnormal operation of peripheral arteries. As a result, arterial lumen becomes narrow or even completely occluded. The early MBTs can effectively promote the recovery of the blood flow of the peripheral arteries, expand the peripheral arteries, and even make them return to normal.

## 5. Conclusion

In the study, 114 patients with severely injured trauma were enrolled into MBT group (67 cases) and NBT group (47 cases) according to whether they accepted MBTs within 24 hours after the admission. They all had bedside ultrasound scanning. The results revealed that early MBTs can elevate survival rate and prognostic living quality and alleviate the atrophy degree of IVC, peripheral artery, and blood vessel of patients with severely injured trauma. Furthermore, bedside ultrasound scanning demonstrated superb capabilities in quantitatively displaying hemodynamics and outcomes of MBTs of patients with severely injured trauma. However, some limitations should be noted in the study. The sample size is relatively small, which may reduce the power and increase the margin of error of the study. A study with an expanded sample size is necessary to strengthen the findings. In summary, the results obtained provide a theoretical basis for the application of bedside ultrasound scanning in diagnosis of patients with severely injured trauma.

## Figures and Tables

**Figure 1:** Comparison of the age and the BMI.

**Figure 2:** Comparison of the hospitalization time and the male ratio.

**Figure 3:** The ultrasound image of a male (aged 34) with traumatic renal laceration caused by a car accident.

**Figure 4:** The ultrasound image of a female (aged 26) with traumatic renal parenchymal laceration caused by a car accident.

**Figure 5:** Comparison of mortality. *Note.*^∗^ indicates that there was a notable difference in contrast with the MBT group (*P* < 0.05).

**Figure 6:** Comparison of IVCE and RVI. *Note.*^∗^ indicates that there was a notable difference in contrast with the MBT group (*P* < 0.05).

**Figure 7:** Comparison of ΔVpeak_L._*Note.*^∗^ indicated that there was a notable difference in contrast with MBT group (*P* < 0.05).

**Figure 8:** Comparison of ΔVpeak_AO_ and ΔVTI_AO_. *Note.*^∗^ indicates that there was a notable difference in contrast with the MBT group (*P* < 0.05).

**Figure 9:** Comparison of ΔVpeak_BA_ and ΔVpeak_FA._*Note.*^∗^ indicates that there was a notable difference in contrast with the MBT group (*P* < 0.05).

## Data Availability

No data were used to support this study.
